The article "The Increasing Centrality of Robotic Technology in the Context of Nursing Care: Bioethical Implications Analyzed through a Scoping Review Approach" was published in 2021. Journal: J Healthc Eng.

# The Increasing Centrality of Robotic Technology in the Context of Nursing Care: Bioethical Implications Analyzed through a Scoping Review Approach

**DOI:** 10.1155/2021/1478025

**Published:** 2021-08-28

**Authors:** Filippo Gibelli, Giovanna Ricci, Ascanio Sirignano, Stefania Turrina, Domenico De Leo

**Affiliations:** ^1^Department of Diagnostics and Public Health, Section of Forensic Medicine, University of Verona, Verona, Italy; ^2^Section of Legal Medicine, School of Law, University of Camerino, Camerino, Italy

## Abstract

At the dawn of the fourth industrial revolution, the healthcare industry is experiencing a momentous shift in the direction of increasingly pervasive technologization of care. If, up until the 2000s, imagining healthcare provided by robots was a purely futuristic fantasy, today, such a scenario is in fact a concrete reality, especially in some countries, such as Japan, where nursing care is largely delivered by assistive and social robots in both public and private healthcare settings, as well as in home care. This revolution in the context of care, already underway in many countries and destined to take place soon on a global scale, raises obvious ethical issues, related primarily to the progressive dehumanization of healthcare, a process which, moreover, has undergone an important acceleration following the outbreak of the COVID-19 pandemic, which has made it necessary to devise new systems to deliver healthcare services while minimizing interhuman contact. According to leading industry experts, nurses will be the primary users of healthcare robots in the short term. The aim of this study is to provide a general overview, through a scoping review approach, of the most relevant ethical issues that have emerged in the nursing care field in relation to the increasingly decisive role that service robots play in the provision of care. Specifically, through the adoption of the population-concept-context framework, we formulated this broad question: what are the most relevant ethical issues directly impacting clinical practice that arise in nursing care delivered by assistive and social robots? We conducted the review according to the five-step methodology outlined by Arksey and O'Malley. The first two steps, formulating the main research question and carrying out the literature search, were performed based on the population-context-concept (PCC) framework suggested by the Joanna Briggs Institute. Starting from an initial quota of 2,328 scientific papers, we performed an initial screening through a computer system by eliminating duplicated and non-English language articles. The next step consisted of selection based on a reading of the titles and abstracts, adopting four precise exclusion criteria: articles related to a nonnursing environment, articles dealing with bioethical aspects in a marginal way, articles related to technological devices other than robots, and articles that did not treat the dynamics of human-robot relationships in depth. Of the 2,328 titles and abstracts screened, we included 14. The results of the 14 papers revealed the existence of nonnegligible difficulties in the integration of robotic systems within nursing, leading to a lively search for new theoretical ethical frameworks, in which robots can find a place; concurrent with this exploration are the frantic attempts to identify the best ethical design system applicable to robots who work alongside nurses in hospital wards. In the final part of the paper, we also proposed considerations about the Italian nursing context and the legal implications of nursing care provided by robots in light of the Italian legislative panorama. Regarding future perspectives, this paper offers insights regarding robot engagement strategies within nursing.

## 1. Background

Since at least the early 1900s, mankind has been fascinated with the opportunity of developing intelligent machines able to act like humans. At the end of a century of technological experimentation, the beginning of the third millennium witnessed a real robotic demographic explosion [1]. In fact, the robotics market has been steadily expanding since the late 1990s-early 2000s. With specific regard to the medical robot industry, in 2012, sales totaled $1.3 billion (1,308 units sold), which increased to $1.4 billion in 2016 (1,600 units sold) and to $2.8 billion in 2018 (5,100 units sold) [2–4]. In 2019, the 7,200 units of medical robots sold drove an estimated industry market value of $2.58 billion. Starting from a value of $5.9 billion relative to 2020, the global medical robot market is estimated to reach a value of $12.7 billion by 2025 [5].

The COVID-19 pandemic is undoubtedly among the key factors driving the growth of this market, in addition to the advantages offered by robotic-assisted surgery (which alone accounts for approximately 65% of the market) and robotic assistance in rehabilitation programs. The pandemic emergency has highlighted the centrality of robotic healthcare to addressing three main needs: to ensure as few human interactions as possible, to quickly and efficiently disinfect large environments (robots capable of emitting UV-C rays, capable of killing almost 100% of viruses and bacteria on surfaces, are widely used), and to replace healthcare personnel exhausted by strenuous work shifts.

Of particular interest for the purposes of this discussion are assistive and social robots, which are employed in a variety of healthcare settings as nursing care providers. According to the U.S. Congress, assistive technology can be defined as “any item, piece of equipment, or product, whether it is acquired commercially, modified, or customized, that is used to increase, maintain, or improve the functional capabilities of individuals with disabilities” [6].

Assistive robots, therefore, represent a special category of robots designed to help patients with disabilities to live independently. Depending on their specific task, assistive robots can be classified into two main categories: service robots and monitoring robots. As regards the first group, service robots can be employed for either mobility assistance or serving and feeding assistance. Service robots with the aim of providing motor support include intelligent wheelchairs and walkers, intended for people affected by lower limb disorders; wearable exosuits for subjects with impaired lower or upper limbs; robotic systems capable of detecting obstacles and intended to help people with visual disabilities to move safely; rehabilitation robots, which constitute an invaluable tool to improve the effectiveness of rehabilitation therapies, helping patients to adequately perform their movements; and carrier robots, which facilitate the process of transferring the patient with motor disabilities from one place to another (for instance, from a bed to a wheelchair) [7].

Service robots designed to provide serving and feeding assistance are particularly common in Japan. They can carry and distribute food trays to patients in care centers and hospitals, thereby substantially reducing caregivers' and nurses' workload [8].

Progress in robotics and intelligent systems allowed to take advantage of robots to provide patients not only with physical and tangible support, but also with intellectual support, in an effort to ensure their psychological well-being and the emotional comfort.

Alongside assistive robots, another category of robots is taking an increasingly central position in healthcare: the so-called social robots.

They are artificial intelligence systems engineered to establish social relationships with humans, being able to relate to them and to engage them with mental activities. They are provided with at least three basic skills: they can focus their attention on the human, creating a bond with the user; they can display social behavior; and they can interact with the environment [9]. Social robots can be further categorized as elder care robots, intended to assist older people; sociable robots that show particularly remarkable interaction skills that enable them to establish strong emotional relationships with humans; and entertainment robots, specifically designed to represent a source of amusement for the user.

As the diffusion of social robots in the healthcare setting is becoming more and more widespread, one of the main challenges we face is the acquisition of technical knowledge to program these agents in such a way that they can act and communicate with patients in ways that are as natural and close to human behavior as possible.

The ever-increasing diffusion of assistive and social robots in healthcare settings is highlighting the relevance of the important ethical issues related to progressive dehumanization in the healthcare context. This dehumanization is, in addition to a series of known issues and already the subject of deep reflection for several years, related to the difficulties of integration of assistive and social robots within the nursing setting. This integration, in fact, must necessarily deal with a theoretical context that must be redefined, or at least updated, since the historical theories of nursing and nursing needs have been developed in a context of entirely human care.

These issues fall within the scope of the topics addressed by medical roboethics, a specific and relatively new research field aimed at identifying the most appropriate way to apply ethical principles and theories to medical robotic applications.

On the cusp of the fourth industrial revolution, medical roboethics is a discipline of central interest, especially in relation to the implications in the nursing field, since assistive and social robots (which are in fact robotic nurses) are now a reality, especially in some countries, like Japan.

Japan has been and continues to be the most fertile ground for the development of robots used in nursing, not only because it is undoubtedly one of the most technologically advanced countries in the world, but also because it is facing a worrying problem related to the ageing of its population [10].

With one of the highest life expectancies in the world, in fact, Japan has a super-aged society: the percentage of inhabitants over 65 years of age is 28.7%, and it is estimated that by 2036 the over-65 population will represent one-third of the population [11].

According to a 2017 forecast by the National Institute of Population and Social Security Research, Japan's population will decline from 127 million in 2015 to 111 million by 2040 and then collapse below the 100 million mark by 2053 and below 88 million by 2065 [12].

This demographic scenario has prompted Japanese authorities to promote healthcare policies increasingly focused on the use of robots as key players in nursing care.

In 2014, Prime Minister Abe Shinzo declared his intention to carry out a real industrial revolution based on the use of robots in healthcare, to complete a strategy of revitalization of the country.

In this sense, Japan is probably the forerunner, since it is highly probable that the path it takes will be followed on a global scale soon.

However, a survey conducted in 27 European countries, also in 2014, showed that more than 50% of respondents expressed strong opposition to receiving care from robots.

In addition, nearly 90% of respondents were uncomfortable with the thought of robots caring for the elderly and for children [13].

In fact, the integration of advanced technological tools so sophisticated that they can interact with patients in the same way as human beings cannot but be accompanied by significant ethical issues, both in general terms and, in particular, regarding nursing care, where the relational aspect plays a pivotal role according to the vast majority of nursing theories.

At the forefront is the aspect of respect for human dignity. As early as the 4^th^ century BC, Aristotle understood that man is a “social animal”; that is, he tends to seek out sociality and interaction with his fellow human beings. Excessive robotization of nursing care runs the real risk of significantly reducing the interhuman relationships of patients, for whom the possibility of interacting with others is very often one of the driving forces behind the development and growth of their moral dimension.

The idea of replacing reference figures for the patient, such as nurses, with mechanical substitutes is in apparent stark contrast to one of the best known and most accepted theories of nursing, the NAC theory (Nursing As Caring), which sees the human relationship as an indispensable means of creating a nursing relationship that is capable of becoming an instrument of care.

With regard to the mother of the theories of nursing needs, Virginia Henderson, it seems complicated to think that the nursing activity provided by robots can fulfil the role of nursing as interpreted by the American theorist and described in her Nature of Nursing: “... to get inside the patient's skin and supplement his strength, will or knowledge according to his needs.”

How can we expect a robot to be able to get inside a person's skin?

Secondly, the extensive use of robot nurses is accompanied by an obvious problem of confidentiality. While nursing robots are nowadays able to exploit complex surveillance systems that can record, store, and transmit countless data relating to the personal sphere of individual patients, this information flow could give rise to privacy violations, which must be prevented through the definition of appropriate healthcare facility regulations and protocols.

Then, there is the central issue of safety of care. Although robotics industry has progressed enormously over the last 20 years in programming skills, we are still a long way from guaranteeing the total and unconditional safety of patients cared for by robot nurses.

Programming failures, communication errors with the artificial interface on the part of nurses and doctors, or simple malfunctions can lead to abnormal behavior of robots and thus put patients' safety at risk.

Finally, there is an issue that affects the whole of the labor sector, not just healthcare, namely, unemployment.

Robots are able to provide high standards of efficiency and productivity, often at a low cost, and are, therefore, likely to lead to a dramatic decline in demand for nursing services provided by real nurses.

In the light of all this, what kind of future should we expect for nurses? Is the fourth industrial revolution really likely to disrupt nursing care, emptying hospital wards of human nurses and replacing them with robots?

The aim of this paper is to illustrate, through a Scoping Review approach, the current scenario regarding the bioethical implications of robotic nursing, summarizing the state of the art of modern nursing robotization approaches with particular reference to their deontological background.

We will also briefly discuss the topic from the perspective of the Italian nursing reality.

Finally, we will propose considerations about the legal implications related to the extensive use of robots in nursing care, with reference to the European and the Italian regulatory context in particular.

## 2. Materials and Methods

The objective of a scoping review is to provide an answer to a scientific question through a thorough analysis of the available scientific literature.

There are several ways to conduct scoping review. One of the approaches that respond most effectively to the needs of a scoping review is undoubtedly that proposed by Arksey and O'Malley [14], who argued that scoping reviews can be implemented to examine the extent, scope, and nature of the literature to identify areas of research where evidence is scarce, to determine the need for a subsequent systematic review, to summarize and disseminate current knowledge, or to uncover gaps and direct future research.

This methodological approach requires the study to be carried out in five phases:

  Step 1: identifying the research questions
  Step 2: identifying relevant studies
  Step 3: selecting studies
  Step 4: charting data
  Step 5: collating, summarizing, and reporting results

In the present work, we used the methodological approach of the Scoping Review in order to provide a comprehensive overview of the current trends regarding ethically efficient integration strategies of robots in the context of nursing care.

We conducted this research not only to outline the state of the art on the topic as it emerged from the study of the scientific literature, but also to identify possible strategies for human-robot integration in nursing care that could be applied in the future.

### 2.1. Identifying the Research Questions

We developed the questions on which this study is based in accordance with the population/concept/context (PCC) framework, suggested by the Joanna Briggs Institute [15].

We decided to base the formulation of the review questions on the methodology outlined by the JBI, as the application of the PCC framework is universally recognized for its ability to optimally respond to the characteristic need of a Scoping Review to address the issue through a more general approach than that of a Systematic Review [16].

We, therefore, identified the PCC strategy as the most effective way of guiding the development of the main and subquestions of the review, recognizing the importance of these being broad in scope.

The primary review question was as follows:

1. What are the most relevant ethical issues directly impacting clinical practice that arise in nursing care delivered by assistive and social robots?
2. Two subquestions then spontaneously emerged:
3. What nurse-led models of care have been developed to combine classical nursing with robot-provided nursing?
4. What are the legal implications directly related to ethical issues referable to nursing care provided by robots?

### 2.2. Identifying Relevant Studies

#### 2.2.1. Databases

We used five databases in this review based on our topic: Ovid Medline, Ovid Emcare, PubMed, Scopus, and Web of Science.

We voluntarily omitted to include databases for searching the grey literature for two reasons.

First of all, given the peculiar specificity and technicality of the topic, we encountered several difficulties in identifying narratives, commentaries, reports, and essays specifically investigating the subject in question. Secondly, in order to guarantee the utmost scientific rigor to the research, we deemed it appropriate to avoid referring to texts with a scientific validity not scrupulously documented.

#### 2.2.2. Inclusion Criteria: The Application of the PCC Framework

Since this study considers the ethical implications of the use of assistive and social robots in nursing in general terms, without reference to a specific population, we did not employ the field “population” as a search criterion.

Regarding the “concept” field, the methodology recommended by the Joanna Briggs Institute suggests including elements that would be detailed in a standard systematic review, such as the interventions and/or phenomena of interest and/or the outcomes.

The phenomenon of interest that is relevant to the purposes of this scoping review is robots and the ethical implications of their use in healthcare; thus, robots and ethical issues became elements of the concept.

Finally, nursing care represents the specific scenario, in which the elements of the concept find their place; therefore, nursing care became the element of the context.

We consciously chose to exclude the context of home care (where, in some countries, assistive and social robots are already widely used) because the care context that this review aims to study is healthcare, and nursing in particular.

For each keyword, we identified several medical subject headings (MeSH) and synonyms to be used as alternative keywords.

Table 1 illustrates the application of the PCC framework to the scoping review question.

#### 2.2.3. Search Strategy

In accordance with the methodological approach recommended by the Joanna Briggs Institute [17], our first step consisted of performing a preliminary search within the Ovid Medline database.

For each PCC element, we introduced the relevant MeSH and keywords, and then we joined the lines related to them to obtain an overall set line for that specific PCC element, combining them with the “OR” Boolean operator.

Finally, we combined all overall set lines with the “AND” Boolean operator, to find the results that addressed all our PCC elements.

We did not set limits in relation to study design or time of publication.

We obtained 930 resulting articles.

Table 2 shows the details of the Ovid Medline search.

We applied the same methodological approach—made the necessary adjustments to keywords and MeSHs—on the databases Ovid Emcare (840 resulting articles), PubMed (970 resulting articles), Scopus (555 resulting articles), and Web of Science (1,256 resulting articles).

Overall, we found 4,551 articles using the above search terms and databases.

We completed the last search on 9 April 2021.

### 2.3. Selecting Studies (Screening Phase)

Once we completed the bibliographic collection phase, we entered the 4,551 articles obtained from the five databases into EndNote software.

The first and preliminary phase consisted of identification through an automatic software tool (and consequent elimination) of duplicate articles (*n* = 2,132) and articles not written in English (*n* = 91).

At the end of the initial skimming procedure, we had obtained a library of 2,328 articles.

Next, we again used an EndNote tool to conduct a first and more superficial screening phase, eliminating articles totally unrelated to the purpose of the review and papers related to implications of technology in healthcare that were not related to the objective of our work, thereby reducing the total number of papers to 545.

We discarded 1,783 articles using an automated system based on automatic title and abstract analysis, as they related to topics that were not relevant to the purposes of this review.

Then, the fourth and the fifth authors read the remaining abstracts independently and eliminated papers that were not useful in identifying an answer to the review questions (*n* = 529), leaving 16 articles for full text review.

The inclusion criteria adopted at this stage were as follows:

1. In-depth analysis of human-robot relationship dynamics
2. Parameterization of the actual nursing bioethics reality according to the main currents of nursing bioethics
3. Presentation of new bioethical perspectives able to combine existing nursing theories with robotic assistance

Specific exclusion criteria for this phase were as follows:

1. Exploration of the ethical implications of nursing care provided by robots, but not with implications related to the context of nursing care (e.g., related to the home care context)
2. Marginality of bioethical implications of the use of robots
3. Provision of nursing care through technological devices other than assistive and social robots
4. Lack of focus on human-robot relational dynamics

All 16 selected papers specifically addressed the ethical implications of the use of robots in nursing, with reference to interhuman dynamics and prospects for human-robot nurse collaboration.

Of the 16 articles, 2 were not available. We read the remaining 14 articles in their entirety and judged all to be suitable for inclusion in the review.

### 2.4. Charting the Data

In order to have the necessary data to answer the review question, we employed a data charting form using the Excel program.

We decided to extract the following data from the selected individual articles:

1. Author(s)
2. Title of the paper
3. Year of publication
4. Author(s)' country
5. Type of article
6. Aims of the study
7. Key findings relating to the scoping review question

The title of the paper allowed us to immediately identify the main focus of the research. The year of publication and the nationality of the authors were useful for understanding the technological (year) and geographical-cultural (country) context that constituted the background to the article.

The indication of the type of article was a fundamental indication for understanding the scope of the study. The aims of the study allowed us to immediately identify the expectations of the researchers and the direction of their research. By means of the key findings, we were able to get an idea of the conclusions reached by the article.

### 2.5. Collating, Summarizing, and Reporting the Results

We reported the results of the research in three different ways: a flow chart illustrating the main stages of the research that led to the results; a narrative summary illustrating in a discursive and synthetic way the objectives of the individual studies and their results; a summary table showing the descriptive elements used in the data charting.

The selected articles can be divided in terms of content into two categories: a first group of papers offering a simple annotated review of the available literature, without advancing proposals for ethical theories of robot integration in nursing, and a second group of papers, within which an actual theoretical approach is instead illustrated to define the role of robots in the nursing setting.

## 3. Results

We used the Preferred Reporting Items for Systematic Reviews and Meta-Analyses extension for Scoping Reviews (PRISMA-ScR) flow diagram guidance [18] to depict the information flow through the several phases of this scoping review (Figure 1).

### 3.1. Descriptive Analysis of Selected Papers

Regarding the first category of articles, those that merely describe the current situation and the scientific evidence on the subject, we essentially found three types of orientations.

A first strand of thought approaches the issue in a substantially neutral manner, highlighting, on the one hand, the unquestionable advantages that an efficient human-robot integration in the nursing sector would bring, but also pointing out on the other hand the numerous obstacles to the realization of this cooperation. It is therefore a position that could be described as intermediate, not overly enthusiastic but not necessarily pessimistic.

Fuji et al. [19] raised the many ethical issues associated with the use of robots in nursing, noting that the relentless and rapid growth of the medical robotics market makes it necessary to outline, as soon as possible, clear strategies for the integration of robots within the nursing context, especially in relation to the patterns of behavior that robots would be required to follow to behave ethically.

However, the author sees the robotic development of nursing care as inevitable and is confident in a fruitful future search for effective solutions to the identified problems.

Christoforou et al. [20] proposed the results of a survey conducted on 115 students of the Department of Nursing, Faculty of Health Sciences, Cyprus University of Technology (CUT).

The questionnaire, administered in the context of the ENDORSE project (a European-funded project aiming to broaden the functional scope of mobile robotic solutions in indoor healthcare settings), was aimed at capturing users' views on the use of robotic solutions in practice.

The questionnaire consisted of six sections: demographics, perceived behavioral control, subjective norm, safety and privacy considerations, operational perspective, and management and financial perspectives.

In general, there was a good predisposition for pairing assistive and social robots with nurses, especially in relation to the more tedious, nonclinical tasks, which respondents saw as easily achievable by robots.

In contrast, respondents highlighted important doubts about the actual applicability of the collaboration between nurses and robots in the clinical field, due to the difficulties in convincing patients and educating new colleagues.

Therefore, from the results of this study, there appear to be excellent prospects for a fruitful collaboration between humans and robots in the nursing context, despite the undoubted existence of critical issues related to users' acceptance of an increasingly less human interaction.

In an interesting review, Servaty et al. [21] attempted to identify the main barriers to and facilitators of the implementation of robotic systems in nursing.

As the outcome of the review of updated literature, the authors identified the following facilitating elements: adapting robot functions to the needs of users; individuals' positive attitude towards technology; positive feelings towards the devices; acceptance of end users (positively influenced by various factors, such as the individuals' possession of computer skills, perceived improvement of quality of care, perceived usefulness of the robot, possession of specific attitudes towards robots, perceived increased independence, etc.); active involvement of healthcare teamwork; considering technology as a source of support for nurses and physicians; and a clear identification of roles, responsibilities, and expectations.

The element that proved to make the integration of robotic systems into nursing most difficult was the nonacceptance of robotic devices by end users, facilitated by a wide range of factors, such as concern that usage of an assistive robot could lead to dependence, unfamiliarity with technologies, concerns about loss of control, fear that personal human interaction would be replaced by actions carried out by robots, fear of decreased social contact, privacy issues, and fear that robots have negative effects on health.

The authors thus identify a substantial balance between facilitating and hindering factors, identifying the proper planning of an effective integration strategy as the element that will define the prevalence of one or the other factor.

A second line of thought that emerged was a rather pessimistic view of human-robot integration in the nursing context.

The authors of the articles summarized below basically see a pretty clear preponderance of elements supporting an integration that is difficult to achieve (or, if achievable, dangerous) compared to elements supporting a future fruitful collaboration between human and robotic nurses.

Metzler et al. [22], for instance, came across as somewhat skeptical about the real possibilities of intelligent automata taking an active part in the nursing care relationship by emphasizing the likely climate of conflict, rather than collaboration, that would be created between human nurses and robots should the latter reach a level of technological advancement, such that they would be able to take an active part in the nursing relationship and not simply execute orders.

Regardless, Metzler identified as a fundamental requirement a real ability of robots to become true companions of the patient, not only able to represent a material support, but able to also fit fully into the relationship of care, the use of AI models based on integrative classical and quantum computation.

Barcaro et al. [23] explored new ways of caring for humans using robotic assistants, considering the ethical issues and questions of respecting human dignity. Specifically, the authors' question was whether there is a possibility that robots will be caregivers capable of preserving moral values and human needs while respecting both the patient and the healthcare professional.

In the researchers' vision, until now, the focus of the answer to this question has been wrongly unbalanced on the patients, being desirable the implementation of an active collaboration between humans and robotic caregivers engaged in the care relationship. From this point of view, robots should be interpreted not as faded copies of humans, but as invaluable resources, in many ways superior to humans, and therefore their diversity should be valued as much as possible.

Finally, the authors identified the dehumanization of robot-assisted nursing care as a serious problem, mainly in the context of elderly care, especially in the light of the fact that, in their view, robots are very unlikely to become moral agents and thus capable of hindering this progressive weakening of human relations.

Robson [24] proposed a vision grounded in the philosophy of Alasdair MacIntyre, a practice-based philosophy that does not propose general theories of what should be done but offers a way of looking at practices and other social structures that allow us to answer the question of what we should do based on the practical experience of contexts.

Robson used a scaffolding of reasoning grounded in the central ideas of MacIntyre's philosophy to test whether robots can perform moral tasks, and, consequently, whether they can perform caring functions.

In Robson's view, since many kinds of social experience (such as the caring relationship between a caregiver and a patient) are essential for moral development, machines, unable to take part in such experiences, can never become moral agents and, therefore, cannot provide care.

Stokes and Palmer [25] also appeared somewhat skeptical about the real possibility of effective inclusion of robots within the nursing relationship.

According to them, no care activity can be totally entrusted to robots, which can, at most, take care of minor tasks, always respecting three main principles: first, robots cannot override the core values of care, i.e., caring; second, robots cannot and should not take the place of human caregivers in performing tasks that can only be completed effectively by humans; and third, robots must maximize the opportunities for the human caregiver to deal with the most delicate and emotionally significant aspects of caregiving.

Then, there is the last current of thought to be found after consulting the literature on the subject, the optimistic one, which is confident that it will be possible to achieve a fruitful and successful human-robot cooperation in nursing.

In the position paper of the Anne Boykin Institute for the Advancement of Caring in Nursing [26], published in 2019, the authors clarified how, even in a care setting where robots take a prominent position, nurses must still always be directly involved in decision-making regarding the design, implementation, and judgement of the use of humanoid nurse robots (HNRs) in healthcare.

The researchers further specified how, concurrent with the evolution of robotics applied to nursing, the development of new theories as the foundation of this innovative type of care will be guided by practice-based and research-based evidence.

In essence, then, the position paper identified nurses as the pivotal professional figures to lead the use of robots in the care setting since nursing care is far more complex than a series of programmable functions.

Grobbel et al. [27] explored the ethical framework of the CCVSD, which is an approach in which nursing practice is the starting point for understanding the impact of the robot on care and thus requires a conversion of the experiences of nursing professionals into elements that can help robot programmers design machines that are increasingly suited to the job they are tasked with performing.

In summary, then, Grobbel and van Wynsberghe's work represents a spur to nurses to take the initiative and define how robots should be employed in clinical practice, since the protection of the sacred nurse-patient relationship and the preservation of ethical patient care represents a moral duty of the nursing professions.

Yew [28] identified care ethics as the most appropriate theoretical framework for solving the many challenges posed using robots in nursing, especially in relation to the care provided to the frailest patients.

Care ethics is a feminist theory based on the principle of interdependence of human beings, arguing that sooner or later everyone needs assistance, thus identifying caring for others as a moral ideal of reference.

In particular, Yew sees as particularly adaptable to the use of robots in healthcare the interpretation that the researcher Joan Tronto gave of care ethics, based on the principles of attentiveness to needs, responsibility, competence, and responsiveness.

Finally, we identified 4 articles by 3 different authors that not only propose a vision of the current scenario and a foreshadowing of future perspectives, but also provide technical elements, based on solid psychological and bioethical theories, to support innovative ethical theories of nursing care at the dawn of the fourth industrial revolution.

Tanioka [29, 30] developed a theory about the ideal approach to take in integrating human nurses and nurse robots, to which he gave the name TRETON.

This is a theory that attempts to bring together the NAC theory with the TCCN theory, which has at its core the transactivity of the relationship between nurse and robot, between robot and patient, and between nurse and patient.

Locsin and Ito [31] proposed an approach called the TCCN theory. This theory is based on four pillars:

1. Persons are caring by virtue of their humanness (a concept borrowed from Boykin and Schoenhofer's NAC theory).
2. The ideal of completeness is a perspective of unity. Therefore, caregivers must focus their care activity on the person as a whole rather than on completing the missing pieces of the patient.
3. The process of knowing the patient has several dimensions and provides for reciprocity.
4. Technological tools must be interpreted and used as tools for care.

Further developing the CCVSD approach, Schoenhofer et al. [32] explored the points of contact between that model and the Boykin and Schoenhofer NAC theory, with the intent of identifying a theory representing an effective synthesis of the two systems.

The syncretic integration of these two systems leads to the identification of three key principles underlying the use of robots in nursing care (constituents of the so-called dance of living caring):

1. The specific setting of application of robotics in healthcare must be based on a dynamic interaction between patient and caregiver (like a dance)
2. A caregiver and cared-for person must reflect each other; i.e., the nurse must conceive of the patient as one who cares for him/her
3. The nurse must hear and respond to calls for caring

The proposed model, in Schoenhofer and van Wynsberghe's opinion, if adopted on a large scale, could facilitate the interpretation of values of care and caring as central elements in setting standards of care for robot engagement in nursing and healthcare.

Table 3 schematically illustrates the main characteristics of the articles under review (author/s, title, author(s)' country, year of publication, type of article, study design (if applicable), aims, and key findings).

The structure of the table reflects the division into two groups of articles described above. For each group, we listed articles in chronological order, from least recent to most recent.

In the light of the findings of a careful reconnaissance of the most significant literature on the subject, we can attempt to provide an answer to the research questions.

The main question was the following: “What are the most relevant ethical issues directly impacting clinical practice that arise in nursing care delivered by assistive and social robots?”

The review identified the current lack of codified bioethical models to define a pattern of effective integration between humans and artificial intelligence in nursing.

Even if, in general terms, the enormous potentialities of a collaboration between humans and automata are well recognized, there is the awareness that the classic model of bioethics of care, known as NAC (Nursing As Caring), is not easily applicable to the context of robotic nursing. On the other hand, there is a general interest in the search for new bioethical models that can support human-robot integration. Some of them have already been proposed, such as the TCCN (Technological Competency as Caring in Nursing) and the TRETON model (Transactive Relationship Theory of Nursing), but they still seem to be far from finding a universal application.

If we consider the other side of the problem, i.e., the willingness of patients to accept robot nursing care, a number of criticisms have also emerged here, mainly related to the feeling of insecurity that the person being cared for sees in robot nursing care.

According to our findings, on the contrary, the issue of a possible violation of patients' privacy does not represent a real impediment, at present, to the implementation of robotic nursing, neither is the issue of occupational shortage, which is an issue not specifically addressed (at least not in an organic and systematic way) within the articles we reviewed.

The first subquestion was as follows: “What nurse-led models of care have been developed to combine classical nursing with robot-provided nursing?”

The most promising nursing models that have been developed to date to enable successful human-robot collaboration are essentially three: the Dance of Living Caring (a combination of NAC and CCVSD models), the TCCN, and the TRETON model.

The features of these models will be described in detail in the following sections.

In summary, we can state that these three models have in common the concept of mutual engagement, intended as the bidirectional attempt to enter into the dimension of others, where the protagonists are, on the one hand, the patient and, on the other hand, the robot nurse and the human nurse. This concept is based on the idea that the introduction of a strong element of technologization within the nursing relationship can represent a means of enrichment of the therapeutic alliance, which does not necessarily conflict with the principles of the classic ethical theories of nursing.

Finally, the second subquestion was as follows: “What are the legal implications directly related to ethical issues referable to nursing care provided by robots?”

Since the articles reviewed were characterized by a strong bioethical slant, we must point out that we were unable to gather significant evidence to answer this second subquestion.

In any case, as far as we could gather from the reading of the papers, the main issue of medicolegal interest related to a robotization of nursing care is represented by the relative legal ambiguity related to the identification of the legal responsible (both from the civil and criminal point of view) of adverse events correlated to robot malfunctioning.

In order to attempt to define this issue more precisely, we carried out an additional literature search electively directed at this topic, which will be discussed in detail in the last section of the paper.

In particular, starting from the European legal context, we attempted to frame the issue in the Italian legal setting, also in light of the interesting theories of the Israeli criminal lawyer Gabriel Hallevy.

## 4. Discussion

### 4.1. Ethical Framework

The leading pioneer in the field of robot ethics, the Italian scientist Gianmarco Veruggio, Director of Research at the Italian National Research Council and Responsible for the Genoa Branch of IEIIT, the Institute of Electronics, Computer and Telecommunication Engineering, coined the term “roboethics” in 2002.

Veruggio gave a precise definition of roboethics [33]: Roboethics is applied ethics whose objective is to develop scientific/cultural/technical tools that can be shared by different social groups and beliefs. Those tools aim to promote and encourage the development of robotics for the advancement of human society and individuals, and to help preventing its misuse against humankind.

The birth of roboethics can be traced back to three main events. The first is the Fukuoka World Robot Declaration (2004) [33], in which three general principles related to human-robot interaction were stated: (1) next-generation robots will be partners that coexist with human beings, (2) next-generation robots will assist human beings both physically and psychologically, and (3) next-generation robots will contribute to the realization of a safe and peaceful society.

The second is the First International Symposium on Roboethics, held in Sanremo (Italy) in 2004 and organized jointly by the Sant'Anna School of Advanced Studies of Pisa and the Theological Institute of Pontificia Accademia della Santa Croce of Rome. The third is the presentation of the Roboethics Roadmap [34], one of the documents produced within the European project Roboethics Atelier, funded by EURON (European Research Robotics Network) and assigned to the School of Robotics of Genoa (Italy).

In the ensuing years, there have been numerous conferences and conventions in the international arena, reflecting the growing attention of the scientific community to the subject.

According to Professor Asaro, a philosopher of science, technology, and media and an expert on issues of technological bioethics, roboethics is called to answer three fundamental questions [35]:

1. How can humans use robots while respecting the principles of ethics?
2. How can humans instruct robots to act ethically?
3. What is the best way to build an ethical relationship between humans and robots?

Corollary queries to the third question are as follows:

1. Is it ethical to create artificial moral agents?
2. How should robots treat people, and how should people treat robots?
3. Should robots have rights?

Although these questions may seem distant from our daily lives, we must take note that, in the coming years, we will live in close contact with robots, humanoid or not.

Hence, what may seem like science fiction now will soon be the norm, just as we are now used to using smartphones and sophisticated cars. It is therefore necessary, as well as ethically advisable, to find from the outset a key to understanding the delicate issues related to coexistence with robots.

Of particular importance, also in relation to the purpose of this review, is the understanding of the ethical implications of the use of assistive and social robots in the health system, which is already a reality in many countries around the world.

However, it is evident that the formulation of meaningful considerations on the matter cannot disregard the determination of a theoretical orientation to be followed since there are countless conceptual approaches to bioethics.

### 4.2. Ethical Theories of Nursing: Is There a Place for Robots?

With specific reference to assistive robots, there are indeed numerous nursing activities robots can already perform or will be able to perform soon: accompanying patients to the bathroom and, more generally, when moving around the ward; allowing for rapid call of the human nurse in case of need; measuring vital signs (body temperature, heart rate, respiratory rate, and arterial oxygen saturation via pulse oximeter); providing body hygiene practices for patients; optimizing bed position of bedridden patients; helping patients feed themselves; lifting patients to measure their weight; administering drugs; automatically adjusting the delivery levels of drugs administered by elastomeric pumps in relation to predefined parameters; automatically adjusting oxygen delivery levels in patients undergoing oxygen therapy; monitoring fill levels of body fluid collection devices (bladder catheter bags, ostomies, drainage bags, etc.); performing simple sampling operations of biological material (urine, feces, sputum); providing close supervision for less autonomous patients; preventing accidental patient falls.

Most of these operations fall within what is known as basic nursing, as defined by some nursing theorists [36]. As for social robots, these interact directly with humans, in a social manner.

In nursing practice, they can be used for mere support activities like reminding patients to take their medication, or they can play a real role in psychological assistance, interacting empathically with the patient and providing emotional support along the care path.

But even assuming that we could have robots capable of performing these tasks, how do we integrate them within nursing care? Which reference model should we adopt (if one already exists) or which new theoretical model should we imagine?

In fact, quality nursing care must be based on a theoretical design that clearly establishes the tasks and roles of the nurse, as well as the dimension that nursing care must take [37].

We begin by describing two of the most important theories of nursing, the NAC theory, which was conceived and designed based on all-human care, and the CCVSD theory, which was created in reverse with the intent of fostering an integration of robotic entities within healthcare.

The NAC theory, postulated by Boykin et al. [38], is based on the pivotal concept that people care for others by virtue of their humanness.

From this basic assumption the principle that caring represents the true essence of living is derived, constituting the full realization of human existence.

Using an eloquent expression from Roach, which encloses the essence of the NAC approach, “caring is the human mode of being” [39].

The nursing care relationship shaped by the NAC model is essentially based on three basic principles:

1. All people are caring, are worthy of respect, and have a role in society
2. Caring is a process that is articulated over time and is strengthened in the relationship with others who care
3. People realize themselves in a specific moment in time, but at the same time, their completeness grows in the caring relationship

In the NAC theory, the context of nursing care is identified as the “shared lived experience in which the caring between nurse and nursed enhances personhood,” to indicate that, within the nursing situation, the nurse enters the world of the person being cared for to get to know the person experiencing care in unique ways, with the intent to grow as a person through the nursing process.

This theoretical framework is flanked by a model that van Wynsberghe proposed in 2015 [40], the CCVSD approach, designed with the intent of paving the way for collaboration between human nurses and robotic collaborators.

The CCVSD theory is based on four fundamental values: attentiveness, responsivity, competence, and reciprocity.

Attentiveness is embodied in the nurse's awareness of the patient's care needs. Responsibility concerns the moral predisposition to bear liability in case of adverse events.

Competence relates to the quality of care provided, which is often intimately connected with the organizational setting of the healthcare facility.

Reciprocity consists of being attentive enough to intercept even the most seemingly insignificant changes in the needs of the person being cared for, to modulate care accordingly.

In the CCVSD model, nursing care does not take on an all-encompassing character, being interpreted more as a response to the needs expressed by the person being cared for, which are therefore the driving force behind care.

The two models have some basic concepts in common (care must be individualized and designed around the specific needs of the person being cared for, and care must be driven by a genuine and intentional desire to get to know the person). They also have three major areas of divergence [41].

First, while the NAC theory is based on the concept of caring, the CCVSD approach is based on the concept of care.

The graphic representation that Boykin and Schoenhofer identified as most representative of caring is the dance of caring persons, the image of five dancers forming a circle, intent on moving freely as individuals listening to music that puts them all in connection with each other.

This image aims to enhance the involvement of all the people involved in the care process, who move forward together, united.

The concept of caring, therefore, has a deep emotional imprint, based on a humanistic ideal, according to which nursing care is provided with a deep and sincere desire to relate to the persons assisted simply because they are human beings.

The concept of care, on the other hand, rather than focusing on the emotional thrust of the nursing care and its objective, is focused on the mode through which this is provided: the care is realized in putting in place a series of activities, which are institutional care practices.

The objective of this approach is to prevent caregivers' conduct from being deemed of quality even in the absence of actual services provided to the cared-for person. To oversimplify, we could say that while caring is based on the reason for and goal of providing care, care is based on how to provide care.

The second element of discordance between the NAC theory and the CCVSD theory is represented by the starting point of the request for nursing care, identified with the call in NAC and with the need in CCVSD.

Boykin and Schoenhofer believed that the call modality represents the best form of request for nursing help, as it minimizes the asymmetry between patient and nurse, which the concept of need tends, instead, to amplify.

Nursing as care theorists reject the idea of need-based care because the concept of need presupposes the existence of deficiencies or shortages on the part of the patient, which require intervention by the nurse (who instead engages in the relationship not to fill gaps in patients, but to know them as a caring person).

On the other hand, according to CCVSD theorists, as well as the interpretations that have been given on the theory, need must be the starting point of nursing, as it must be interpreted from the perspective of the concept of care, thus the implementation of specific and highly specialised nursing practices.

From this point of view, therefore, the concept of need should not refer to the concept of vulnerability of the person assisted but should focus on the omnipresence of the needs of the assisted, which an adequate activity of care must be able to satisfy.

Finally, the third element of discordance between the NAC and the CCVSD theories is the source of value priorities, identified in the ideal of the dance of caring persons by the former and in the hospital institution by the latter.

In fact, as is evident, while the NAC approach sees its value foundation in the reciprocity of therapeutic assistance, the CCVSD approach sees in institutional efficiency the main source of those care practices indispensable to respond to the patient's needs.

Having dealt with the essentials of the two models, it is time to ask whether these models are applicable to robot-delivered nursing care. Evidently, the CCVSD model is much closer to an approach that can facilitate effective placement of robot nurses, and it is no coincidence that it was designed 14 years after the NAC model, thus in a profoundly changed technological context. The CCVSD model was conceived with the intent of studying a system that would facilitate the integration of technology into nursing care.

The concept of care (as illustrated), emphasizing the centrality of the response to the needs of the patient and a value system identified in the efficiency of the health institution, is in fact much more compatible with nursing care that is less human but in some ways more efficient.

However, we cannot exclude the hypothesis that the approach based entirely on CCVSD theory runs the risk of excessively dehumanizing nursing care by not incorporating some of the key principles of the NAC theory.

It is with a view to optimizing the CCVSD approach that the theorists of the two paradigms (Schoenhofer et al.) formulated in 2019 a new joint proposal for a vision of nursing, enriching the CCVSD model with the values of the NAC model, arriving at a theory that they called the dance of living caring, which represents for them the best possible strategy to guide the engagement of robots in nursing care [42].

The graphic representation of the dance of living caring is identical to the scene of the five dancers in the dance of caring persons, but with the difference that one of the five dancers is a robot. This means, in essence, that the new theory attempts to find an effective synthesis between the NAC model and the CCVSD model, enhancing their respective strengths.

In practical terms, the theory of the dance of caring living is based on three key principles:

1. Intentional knowing of persons as caring (which adapts the NAC principle that each person is recognized as caring and the CCVSD's concept of coming to know the assisted person)
2. Respecting and valuing persons as caring (which blends the NAC principle of a relational care process and the commitment to reciprocal engaging concept of CCVSD theory)
3. Responding to calls for caring (which brings together the responding to what matters of the NAC theory and the providing effective responses to needs of CCVSD theory)

In essence, the dance of living caring model represents the theoretical substrate for ensuring that nurses can have robots participate in the caring process in a manner that is instrumental to the pursuit of an ethically virtuous caring relationship.

In the dance of living caring model, in fact, the choice of whether to introduce and when to introduce robots into the caring relationship occurs through a dance, a shared pathway between nurse and caregiver.

Another interesting theory that attempted to adapt the NAC theory to the technological advancements of the fourth industrial revolution is Locsin's theory of TCCN [43].

This theory proposes to enhance the technological evolution as an element that allows nurses to ensure an even better quality of care relationship, starting from the concept that technology can bring the patient closer to the nurse.

According to the TCCN theory, the caring relationship is based on three pillars: technological knowing, which is basing one's knowledge of the other on revelations from technology; designing, which is that multidimensional process such that both the nurse and the person being cared for work together to create a mutually satisfying process of care that the nurse employs to deliver quality care to patients to meet their needs; and participative engaging, which involves the nurse and the person being cared for simultaneously practicing shared activities that are intended to ensure that they know each other.

In other words, according to the model Locsin proposed, technological competence as care in nursing represents the use of technology to enter more effectively into the dimension of the care recipient, and, in so doing, understand more accurately the care demands of patients and respond accurately and appropriately to their needs.

In summary, therefore, Locsin presents an unprecedented view, conceiving technological competence as a fundamental element in nursing care, since the knowledge of technological tools demonstrates the attention that the nurse pays to the persons assisted, to be understood as collaborators in their care rather than objects of their care.

Another of the important modern theories of robotic integration in nursing is the one Tanioka formulated in 2017, which attempts to merge the NAC approach with the TCCN approach; this is the TRETON [44].

This is an innovative theory that has at its core the transactivity of the human-robot relationship. That is, the nursing process becomes a transactive engagement based on the nursing encounter, which corresponds to the nursing situation that Boykin and Schoenhofer described in the NAC theory.

The adaptation of the NAC theory to nursing with robots as the central characters causes technological knowledge to become a crucial dimension, representing the initial stage of knowing.

From TCCN theory, TRETON theory takes the concept of mutual engagement, which in Tanioka's theory becomes the context within which the transactional relationship occurs.

Such mutual engagement, which provides that the nurse, the robot, and the patient may passively or actively participate in creating a plan of care, is complemented by a technological engagement, which consists of the transactional relationship between robot and patient, the process by which the robot enters the dimension of the assisted.

The ability of nurse robots to enter the world of patients and thus to know them is the cornerstone of nursing care delivered by HNRs, and can be achieved through four patterns of knowing:

1. Empirical knowing: this is accomplished through the ability of HNRs to access databases and the Internet, through which robots can learn the entire medical history of the person being cared for and then communicate it to the human nurse.
2. Aesthetic knowing: this takes the form of the HNRs' ability to store and archive data about patients' wishes and emotions as well as to accumulate personal data such as photographs and lab data, which can be made available to family members at the most opportune time
3. Personal knowing: this relies on the robots' ability to collect and store the data they detect on a day-to-day basis (vital parameters, patient's physical condition, patient's emotions, etc.)
4. Ethical knowing: as discussed in the previous section, there are currently no well-defined standards to guide the ethical choices of robots, relying for now on rudimentary ethics education systems that are likely to be implemented effectively in the years to come

Thus, TRETON theory represents a highly effective paradigm for the inclusion of robots in nursing: the occurrence of nursing encounters involving human persons and HNRs represents an extraordinary driver for the implementation of transactive engagement, which may soon form the basis for the systematized and extensive use of robots in nursing.

The only perplexity that arises is this: if HNRs can demonstrate full technology in nursing, what will make them different from the nursing expertise displayed by current human nurses?

Another well-known ethical theory of nursing that deserves to be explored is the ethics of care theory. Ethics of care (or care ethics) is a contemporary ethical theory based on the principle that it is ethically correct to put the interests of those close to us before the interests of those not emotionally connected to us.

It is therefore clear that the scenario of care ethics is in sharp contrast with ethical theories based on principles that aim to highlight moral actions, such as Kantian deontology, utilitarianism, and the theory of justice, and does not intend in any way to be incontrovertible and take on the character of axiom.

Care ethics can be declined essentially according to three interpretations: that of Tronto, that of Held, and that of Vanlaere and Gastmans. Tronto [45] identified four decisive elements in the caregiving process: attention (or awareness), taking responsibility for the patient's needs, competence (not only professional, but also in terms of empathic skills), and the patient's personal emotional response to the care provided by the caregiver.

In Tronto's conception of care, AI may only superficially satisfy some components of care, but not all. Indeed, no matter how efficient the robot may be in assisting the patient, it can never have a level of understanding of the needs of the subject it is assisting that provides it with an ethically relevant awareness of those needs.

According to Held's interpretation of care ethics, the caring practice shows us “how to respond to needs and why we should. It is not a series of individual actions, but a practice that develops, along with its appropriate attitudes” [46].

In essence, then, according to Held, care presupposes that individuals are interpreted as relational and interdependent beings. Furthermore, Held argued that the caring relationship and trust represent two distinct, albeit intimately related, concepts, as both are essential to the maturation of interpersonal relationships.

Regarding the inclusion of assistive and social robots within nursing, according to Held, because the nursing relationship is a reciprocal and interdependent social relation between patient and caregiver, machines equipped with AI are automatically excluded from taking part in that relationship.

Regarding the connection between the concept of caring and trust, AI, while being able to imitate and reproduce some human actions capable of arousing trust (and trust is to all intents and purposes a moral concept), is not able to field a moral attitude.

Also, the concept of trust implies the concept of betrayal, and it is objectively very difficult to think that a machine equipped with AI can betray a human, as it is not equipped with a moral sense.

Vanlaere and Gastmans [47] argued that care ethics should be thought of through a personalist approach, in the belief that people provide care to other people because failure to do so diminishes the personal fulfilment of the potential caregiver and the care recipient.

In Vanlaere and Gastmans' view, caregiving concerns should be entirely focused on attention and the ability to tune in to the other person's emotions. In this view, it is critical that the caregiver act responsibly, given the vulnerable nature of the persons being cared for.

Even in Vanlaere and Gastmans' view of care ethics, AI does not have the elements to fit into the caring relationship, since robots, no matter how advanced, do not possess an emotional intelligence equivalent to that of humans.

### 4.3. The Nursing Need Theories: Can Robots Meet the Needs of the Assisted Persons?

Concurrent with the evolution of medical science was a contextual understanding of the centrality of nursing care as an integral part of the nursing relationship.

This awareness has led to the need to define, in an organized and systematic way, the needs of the patient to whom nursing care should be directed.

There are six major nursing need theories on which the nursing care relationship is based, which we will summarize to identify possible spaces for the inclusion of assistive and social robots.

Marjory Gordon's model is based on the principle that all-human beings share certain functional patterns that contribute to their health, quality of life, and realization of human potential.

These common patterns represent the focus of nursing assessment.

By the term “pattern,” Gordon means a group of behaviors that are repeated cyclically over time; the continuous interrelationship between these goes to determine the complexity of an individual [48].

The 11 patterns Gordon identified, and on which nursing attention should therefore be focused, are health perception/management pattern, nutritional/metabolic pattern, elimination pattern, activity/exercise pattern, sleep-rest pattern, cognitive-perceptual pattern, self-perception/self-concept pattern, role/relationship pattern, sexuality pattern, coping pattern, and value/belief pattern.

Certainly, best known is the model of Virginia Henderson, one of the world's most famous contemporary nurses. In Henderson's vision, the primary objective of the nurse must be to assist individuals (healthy or ill) in performing those activities that contribute to their well-being, activities that they would perform independently if not provided with the necessary will, strength, or knowledge.

In other words, therefore, the nurse must ensure that the assisted person achieves or regains a state of independence as soon as possible [49]. In the metaparadigm that Henderson theorized, the person represents the entity in need of assistance, health is identified in the autonomy of the person in the management of their health needs, while nursing is the support activity provided to subjects to ensure the possibility of recovering their autonomy.

There are 14 individual needs that Henderson identified as essential: breathing normally; eating and drinking adequately; eliminating body wastes; moving and maintaining desirable postures; sleeping and resting; selecting suitable clothes—dress and undress; maintaining body temperature within normal range by adjusting clothing and modifying environment; keeping the body clean and well-groomed and protecting the integument; avoiding dangers in the environment and avoiding injuring others; communicating with others in expressing emotions, needs, fears, or opinions; worshipping according to one's faith; working in such a way that there is a sense of accomplishment; playing or participating in various forms of recreation; learning, discovering, or satisfying the curiosity that leads to normal development and health; and using available health facilities.

Another authoritative nursing need theory is that of Dorothea Orem, the so-called self-care deficit nursing theory. According to Orem, the driving force behind the request for nursing care is represented by the existence of a deficit of self-care, such as to make individuals unable to perform autonomously those actions that allow them to preserve their well-being.

Orem's model finds application primarily in rehabilitation and primary care settings, and generally in all areas of healthcare where patients are spurred to achieve independence. According to this theoretical model, in fact, all of a patient's self-care behaviors represent a decisive boost to the achieving recovery.

If a patient is unable to implement self-care, a self-care deficit is realized, necessitating the intervention of the nurse, who can act through three modes of intervention of increasing intensity: fully compensatory, partially compensatory, and supportive/educational [50].

Then, there is the well-known theory of Peplau, strongly centered on a psychodynamic model and defining the nursing relationship as based on the exploration and management of the psychological meanings of the patient's values, feelings, and behaviors [51].

Specifically, Peplau's model envisions that the care relationship is articulated in four distinct phases: orientation, in which the nurse and patient work together, so that the patient faces the condition of illness/discomfort in a positive spirit; identification, in which patients attempt to become aware of their real possibilities for resolving their situation; development, in which nurse and patient plan together the goals to be achieved and patients mature to the idea that they are capable of self-care; resolution, in which the relationship between patient and nurse becomes less and less close, with a gradual attenuation, until extinction, of the identification process.

The nurse can assume six roles in the care relationship: stranger (at the beginning of the therapeutic relationship), resource (the healthcare provider is seen as the one who can meet the needs of the patient), educator (the nurse teaches patients to use their state of disadvantage as a source of enrichment), participatory leader (the nurse acts by supervising and coordinating the patient), substitute (the patient identifies in the nurse a series of emotions felt in the past), and consultant (the caregiver represents the person with whom the patient can share his or her state of mind).

A theory with a holistic view to the discipline of nursing is Madeleine Leininger's theory of transcultural nursing. Leininger's model is, in fact, built from a set of multiple elements: the social structure, the worldview, the values, the environment, the language, and the professional systems of the society, in which one is going to act.

According to Leininger, care is a universal phenomenon, which must be inserted into the cultural setting, in which it takes place. In fact, the care of oneself and others changes profoundly in different cultures and different systems of care.

Nurses, in their practice, must therefore take intercultural data into account. It will follow, for example, that highly technologized care will not always be able to meet the expectations of assisted persons who are not open to technology [52].

Finally, we report a nursing need theory particularly appreciated in the Italian healthcare context, the model of Marisa Cantarelli, the first Italian nursing theorist.

In Cantarelli's vision, people, in conditions of normality, can interact in their environment, satisfying their needs in autonomy and thus preserving their state of health.

If conditions that disturb this balance arise, someone must take over to assist the subject. However, this assistance, which can be provided by anyone at a first level, at a certain level of need, can only be provided by professionals with specific skills.

In the case of needs involving the person's body or psyche, the nursing professional can legitimately respond to the specific needs of nursing care [53].

The theory in the nursing performance model identifies 11 nursing care needs: need to breathe, need to feed and hydrate, elimination needs, need for hygiene, need for movement, need for rest and sleep, need to maintain cardiovascular function, need for a safe environment, need for interaction in communication, need for therapeutic procedures, and need for diagnostic procedures.

For each need, there are 11 actions of nursing care, defined as “performances,” i.e., the results achieved through the performance of a complex of actions coordinated with each other, to resolve a specific need manifested in a patient.

According to Cantarelli, the activities performed by the nurse are, in ascending order of care complexity, addressing, guiding, supporting, compensating, and replacing.

Having outlined the theoretical framework of care needs to be met by nursing, can robots respond to one or more of the models?

On closer inspection, there do not seem to be insurmountable obstacles to the possibility of robot nurses adhering to the nursing need theories illustrated.

Taking Henderson's model as an example, according to which “the unique function of the nurse is to assist the individual, sick or well, in the performance of those activities contributing to health or its recovery (or to peaceful death) that he would perform unaided if he had the necessary strength, will or knowledge” [54], a robot could easily respond (in some cases even more effectively than a nurse) to needs that would allow individuals to regain their autonomy as quickly as possible.

The same considerations can be extended to the other models described, except, perhaps, for Peplau's model, which, in addition to providing a definition of nursing needs, proposed a strongly human connotation of the nursing relationship, considering nursing as a “significant, therapeutic, interpersonal process.”

Peplau's theoretical framework, therefore, seems difficult to reconcile with totally dehumanized nursing care.

However, if we consider, for example, Leininger's approach of transcultural nursing, it is evident that the participation of robot nurses represents an extraordinarily advantageous support to achieve the encounter between cultures that the theorist desired.

Consider the language aspects: what better cross-cultural adaptation in nursing than interaction with a social robot that can speak a foreign language with the patient?

Therefore, the transcultural nursing model seems to be perfectly adaptable to robotic nursing care, facilitating in a decisive way the encounter between the cultures of the actors in the nursing relationship.

There remains the problem, mentioned earlier, of the adaptability of Leininger's model to subjects not ready to accept the technology, a problem difficult to solve, in fact, but that on closer inspection could be overshadowed by the benefits, in terms of cultural rapprochement, that the use of a robot could bring.

As for Cantarelli's and Orem's models, they are in many ways close and characterized by the same concept of need—the individual's necessity to receive nursing care when certain mental or physical conditions occur that require it—having the individual as the focus of interest (as well as many other nursing need theories that we did not discuss, such as the theories of Nightingale, King, Neuman, and Rogers), and therefore they seem well suited to robot-delivered nursing care.

In fact, efficiency in terms of timely and appropriate response to the needs of the individual seems to be precisely the strength of robots, which would therefore have no difficulty in ensuring adherence to such models of care.

The problem related to the ethicality of this relationship is a completely unrelated issue and should be assessed by separating it from the evaluation related to the ability to meet the needs of the assisted.

In other words, a robot nurse could fit perfectly within the theoretical context of a nursing need theory (e.g., Leininger's theory), but it would not fit within the ethical framework of the ethical theory of nursing that one decides to adopt.

Therefore, we must always keep in mind that when evaluating the role of robots within nursing, the two theoretical frames of reference, that of nursing needs and that of the ethical relationship, must be clearly distinguished.

### 4.4. The Evolution of Ethical Design from Asimov to Modern Roboethics: Teaching Robots to Behave Ethically

The term “ethical design” refers to the process, by which a high-tech product is instructed to implement ethically appropriate behaviors.

The process can be achieved through two approaches: top-down or bottom-up. In the first case, a code of ethics is introduced into the system and incorporated into the robot's algorithm, while, in the second case, the robot implements a machine learning process based on the observation of human beings and the ethical values they put into practice.

The first model of ethical design dates to the 1940s, when the American writer and biochemist Isaac Asimov devised the well-known Three Laws of Robotics, developed with the goal of establishing theoretical principles for his robot-based fiction.

The three laws represent a rudimentary robotic ethical system, with a strong human-centered vision.

The principles, first illustrated by Asimov in the science fiction short story “Runaround” in 1942, read as follows [55]:

1. Law 1: a robot may not injure a human being, or, through inaction, allow a human being to come to harm
2. Law 2: a robot must obey the orders given it by human beings except where such orders would conflict with Law 1
3. Law 3: a robot must protect its own existence as long as such protection does not conflict with Laws 1 and 2

Later, Asimov added a fourth law, called the Zeroth Law, more important than the previous ones, so named to go on with the pattern, according to which lower-numbered laws take the place of the higher-numbered laws, which read as follows: “Law 0: no robot may harm humanity or through inaction allow humanity to come to harm.”

Asimov's intent was clear: through the setting of the four laws, he tried to lay the groundwork for definitively overcoming the Frankenstein-like plots in science fiction literature, in which man was invariably forced to destroy robots to protect mankind from their destructive potential [56].

The main weakness in Asimov's concept of human-robot relationship lies in assuming robots to be in possession of sufficient decision-making autonomy to allow them to make moral judgements in every possible situation, regardless of its complexity.

In other words, Asimov's three laws would be virtually applicable only if robots are equipped with a highly developed AI, a condition existing in the author's science fiction stories (where robots were equipped with positronic brains) but very difficult to apply to reality [57, 58].

In the early 2000s, with the explosion of the robotics industry, there was a concomitant need to reevaluate and modernize the four laws, which were universally believed to be difficult to apply in practice.

The increasing diffusion of robots gave, therefore, a strong impulse to the birth of a discipline aiming at defining a code of ethics suitable for a world where human beings and robots coexist.

In fact, it seems clear that Asimov's laws, although they undoubtedly represent an evocative starting point, at present cannot be of any practical use in the formulation of propositional reflections and need to be revisited.

For example, the researcher Fedaghi proposed to reformulate Asimov's laws by applying to them a classification scheme of ethical categories, with the intent of simplifying the process through which the robot should select the most ethically correct action to put into practice [59].

According to Fedaghi's vision, an “ethical category” represents an ethical context that comprises a typified moral agent and a moral patient.

The typified moral agents can be human agents, organization agents, or artificial agents (including robots). The typified moral patients are categorized as human patients, human-based organization patients, and artificial patients. There are therefore nine possible combinations of moral agents and patients.

Every moral agent and every patient can be characterized by three values: good, evil, or neutral. This results in a taxonomy consisting of as many as 81 combinations, which correspond to the ethical categories, 45 of which are the domain of artificial agent ethics.

Fedaghi's intent, through this categorization system, is to make it easier for the robot to choose the most ethically correct conduct, even in the most complex situations, bringing the concrete situation into one of the established ethical categories.

Obviously, the selected ethical values (good, evil, or neutral) simply represent one of the most common classifications of ethical principles, proposed by the author for reasons of expositive clarity, since the suggested system can be adapted to any other classification (for example, if, instead of three ethical values, we take four, the ethical categories would be 169).

Fedaghi then offered a new key to reading Asimov's laws, which he reformulated by integrating them with the system of categorization of ethical situations he proposed, in accordance with the principles of procedural ethics, which aims to develop procedures capable of guiding the process by which ethical decisions are made [60].

Another interesting approach, and in many ways like the one described above, is the one Professor Selmer Bringsjord, of the Rensselaer Polytechnic Institute, proposed, which draws inspiration from the so-called dream of Leibniz [61]: the desire to devise a symbolic calculation, an algebra of thought, that would solve any kind of problem.

According to Bringsjord's vision, the foundation on which the ethical reasoning of robots must be based should not be represented by Asimov's laws, but by deontic logic, a discipline opposed to classical logic that employs particular logical operators to formalize an ethical code [62].

In other words, Bringsjord proposed a general methodology, based on deontic logic, with the aim of making robots follow certifiably ethical conduct.

Certification of the ethical correctness of the robot's behavior would be verified through two formal proofs, which establish two conditions:

1. Robots can only perform permissible actions
2. All actions that are mandatory for robots are performed by robots themselves (influenced by ties and disputes among the available actions)

In Bringsjord's view, the approach based on logic turns out to be best, as the use of mechanized formal proofs appears to be the only suitable tool for the determination of a solid relationship of trust between man and robot [63].

An approach that differs sharply from Fedaghi's and Bringsjord's is case-based reasoning (CBR), which is based on the idea that one can behave ethically even without having learned any notion of ethics.

In fact, CBR is a mode of reasoning by analogy, which aims to find solutions to new problems through the analysis of solutions to similar problems that have previously arisen. Many researchers have developed computer systems capable of processing (and in some cases putting into practice) moral principles and precepts based on a CBR mechanism.

Of particular interest, for example, is the experience of Iranian researchers Honarvar and Ghasem-Aghaee [64], who employed a CBR strategy to instruct an artificial neural network to perform a classification of what is or is not ethically correct.

Utilitarianism represents another possible theoretical approach to interpreting machine ethics. Utilitarianism takes as its starting point the affirmation that it is a condition of human nature to think first and foremost of one's own interest. According to utilitarian logic, morality consists in recognizing that the individual's greatest usefulness coincides with the usefulness of others.

The utilitarian approach, although easy to implement, is very difficult to apply in practice, since it poses a serious risk to the fundamental rights of the individual. In the utilitarian logic, in fact, activities such as killing, stealing, enslaving, and mistreating can be considered ethically acceptable in certain circumstances, as in cases where they bring an advantage to the community (think, for example, the killing of an evil person hated by all) [65].

A further orientation is the rule-based system that Powers proposed. Powers started from the assumption that a code of ethics can be translated into a set of practical rules. The application of a rule-based system to robotics allows robots to mimic human intelligence, inferring new ethical precepts applicable to specific practical contexts from a general theoretical framework.

In Powers's view, the ethical system from which the robots derive the general principles for the formulation of rules would be the Kantian categorical imperatives, chosen because they offer a computational structure for judgement [66]. However, Powers's approach has not been spared harsh criticism on the grounds that the use of machines as implementers of Kantian ethics would be at odds with Kantian ethics itself, according to which moral agents are both rational and free (whereas machines can only be rational) [67].

In light of the above, there are many attempts to introduce within the robotic intelligence a sort of code of ethics able to guide the machine in its decisions. However, if it could be realized, the integration of a moral conscience within an AI would raise a long series of problems, not only of an ethical nature. For example, there would be a real risk of an excessive simplification, even trivialization, of moral precepts. But even more serious risks could be looming, for instance, an extensive and massive use of robots might risk a take-over from humans if not properly controlled.

This is the opinion of Vanderest and Willems [68], who proposed to abandon the idea of basing the decisions of robots on standardized philosophical models, and to adopt instead an empirical approach to the selection of moral precepts that a robot is called to follow.

These researchers administered an online questionnaire to 304 subjects aged 19 to 67 years, mostly working in neither healthcare nor research, with at least a high school education. In the first part of the questionnaire, respondents ranked two sets of actions based on the level of violation of patient privacy or autonomy. In the second part, subjects indicated which actions potentially causing patient distress they felt were permissible in different scenarios.

Of the 304 subjects enrolled to complete the questionnaire, 223 performed the additional task of ranking robotic actions according to their impact on the patient's autonomy and privacy. Overall, the survey showed that the data obtained from the research have characteristics that make them suitable to be translated into a series of operational indications that guide robots in their actions, thus opening the doors to a possible new frontier in the field of ethical decision-making of robots.

### 4.5. The Implications of the Use of Assistive and Social Robots in Nursing Care in the Italian Ethical Perspective

Since social and assistive robots will perform purely nursing roles, it is particularly interesting to analyze the code of ethics of Italian nurses, to identify any critical issues in the flanking of human operators with robotic colleagues.

The first code of ethics for Italian nurses dates back to 1960, six years after the establishment of the Professional College of Nurses, Health Care Assistants and Child Care Supervisors (IPASVI).

The principles were taken from the precepts of natural moral law, a concept borrowed from the philosophical current of natural law. In this perspective, the patient was considered as a subject in a state of disadvantage secondary to the condition of disease, and therefore to be protected through the implementation of protective measures (in line with the modern concept of advocacy).

Seventeen years passed before the nursing profession provided a renewal of the deontological code (in 1977), made necessary by the profound cultural, social, and economic changes and health needs that led, in 1978, to healthcare reform with Law 833, instituting the Italian National Health Service.

The second version of the code of ethics provided for the concrete adherence to the rights enshrined in the constitutional charter, including the right to health, which reflects a renewed conception of the human being.

The third version of the code of ethics, in 1999, reflected a cultural, social, and professional situation that evolved very rapidly from that point.

The code, introduced by the 1996 Nurse-Citizen Pact, addresses new issues that previous versions had not dealt with, such as direct responsibility for nursing care, conflict between values and recourse to conscientious objection, direct references to areas of professional practice, continuing education and updating of knowledge, rules of conduct in emergency situations, respect for the wishes expressed by the person being cared for, concept of restraint measures as an extraordinary event, protection of minors, organ donation, responsibility in compensating for organizational deficiencies, and interaction of the professional with the professional college.

Ten years later, in 2009, the fourth draft of the deontological code of nursing professions was born, in which it was possible to clearly read the will to emphasize the evolution of the rights of citizens and assisted persons in the field of health and life cycles (from birth to death). It considered the assisted person the bearer of all the rights of citizens, in any condition.

The fifth and most recent version of the code of ethics for the nursing professions was approved by the National Federation of Orders of Nursing Professions (FNOPI) in April 2019.

This brief history, illustrating the temporal evolution of the Italian nursing code of ethics, aims to highlight how the ethical precepts applied to the health sector, which are often mistakenly seen as immutable, frequently need to be reviewed and updated, in relation to the evolution of customs and society [69, 70].

Reconnecting to the subject of this discussion, we consider whether the current nursing code of ethics is sufficiently up to date to be applied to care that sees human health workers flanked by assistive and social robots.

Before answering this question, we reflected on the latest version of the Italian deontological code, the 2019 version.

There is a consolidation of the principle of self-determination of the person assisted and the principle of full professional responsibility of the nurse during the entire duration of the care process.

These changes must be primarily ascribed to the novelties introduced into the judicial system by two important laws, Law 24/2017, reforming health professional liability, and Law 219/2017, introducing the living will.

One of the most interesting innovations that we can find in the 2019 version of the Nursing Code of Ethics is borrowed precisely from Law 219/2017, which, in addition to introducing the living will, makes numerous firm points about informed consent, establishing that “the time of communication between doctor and patient constitutes time of care.”

This concept is taken up in Article 4 of the deontological code:

Article 4 (Care Relationship)

In his or her professional activities, the nurse establishes a relationship of care, using listening and dialogue. He/she ensures that the person assisted is never left in abandonment, involving, with the consent of the person concerned, his/her reference figures, as well as other professional and institutional figures. Relationship time is care time. [71].

That seems to be the focus of the robotic turn in nursing.

Should the awareness of the absolute centrality of the human relationship with the person assisted, which is substantiated also and above all with communication, which becomes an integral part of the care, see in the next advent of robots to flank nurses a threat or a possibility of enhancement?

If by communication we specifically mean verbal communication, all the requirements seem to exist to be able to be confident in a communicative dimension not hindered but strengthened by robotic technology.

Consider, for example, the telemedicine services that nurse robots can provide.

In fact, robot nurses hosting telepresence platforms represent an extraordinary tool to implement remote communications between patients and physicians.

Communication as care time is clearly enhanced and valued by such use of robotic technology.

Consider, more simply, the new dimension of the simple communication of the clinical status to the patient through the support of a robotic nurse able to illustrate through a monitor the details of the clinical condition, for which the patient is treated (presentation of the pathology through short videos, explanation of therapeutic approaches, the probability of success of the same, etc.).

Alternatively, imagine presenting a patient with a complex surgical procedure using a robotic nurse that projects a film or creates a hologram illustrating the anatomical structures in real size.

These simple examples demonstrate how robotic accompaniment can represent for nursing care an extraordinary means to fully realize the communication phase of the therapeutic process, identified as crucial in the last version of the Italian code of ethics.

However, there is more than just verbal communication.

Take human contact: despite being a true form of communication, the existential impact of touch in the nurse-patient relationship is often overlooked.

According to some scholars, clinical information communicated through contextual human contact is received very differently than the same information communicated only through language.

This is because it is now clear that physical contact between nurse and patient acts as a channel that can convey messages more effectively [72].

Communication between nurse and patient, in addition to human contact, finds another decisive support in empathy.

Beddoe and Murphy defined empathy as “… the capacity to understand and respond to client's emotions and their experiences of illness” [73].

Communication without empathy is severely lacking, and to the question of whether robots can feel empathy, we are all inclined to answer in the negative, at least for the moment.

“For the moment” is appropriate, since a recent experiment conducted at Columbia University in New York has certified that the road to robotic empathy is now marked [74].

In the experiment, a very simple robot with AI was able to predict the behavior of another robot simply by observing it.

This is the first sign that even in robots could exist a theory of mind, that is, the ability of primates and humans to identify with each other to predict their actions.

We can therefore conclude that, at present, it seems unlikely that the relationship time referred to in the Nursing Code of Ethics can achieve the fullness of communication, assuming the characteristics of real care time, in a relationship exclusively between robot nurses and patients; however, there is reason to expect a change of this kind soon (there are very good conditions for designing robots that are able to feel empathy).

Another interesting passage in the above code (the current version) is Article 36 (Support Workers):

“The nurse, at the various levels of clinical and managerial responsibility, plans, supervises and verifies, for the safety of the patient, the activities of the support workers present in the care process and entrusted to him/her.”

This provision, contained in Chapter VI (Organization) and absent in the previous version of the text (2009), although not directly mentioning robots, seems to apply to a care setting in which the nurse plays the role of supervisor and guide of a robotic collaborator.

Even in the case where the postulate referred exclusively to physical persons (specifically, social-health workers, specialized auxiliaries, or technical operators in charge of assistance), its formulation makes it perfectly adaptable to a context of human-robot collaboration. Given the current impossibility of envisaging nursing care provided exclusively by robots, the supervision of robots by nurses is of crucial importance.

A final aspect to highlight is the focus reserved by the 2019 code of ethics on communication aspects in Article 21 (communication strategies and modes):

“The nurse supports the relationship with the person being cared for who has conditions that limit their expression, through effective communication strategies and modes.”

This article is included in Chapter IV (Relationships with patients) and deals with the issue of communication with the patient in a much more profound way than the similar article in the previous version of the text (Article 24: “... adapting communication to the patient's ability to understand...”).

In the 2009 version of the code, in fact, it seems that the nurse's task is limited to the use of language appropriate to the level of schooling and education of the patient, while in the latest version of the code there is a generic reference to conditions that limit expression, which are not only cultural but may be directly related to a disability.

This extension of the concept of communicative adequacy also seems to be affected by the influence of the increasing technologization of care, which can overcome communication barriers that a few years ago seemed insuperable.

It is exactly in this frame that social robots can be most useful. With their peculiar communication skills, they represent the ideal tool to fill the communication gap between nurse and assisted person.

### 4.6. Legal Implications of Robot Use in Nursing: Food for Thought about the European and Italian Regulatory Context

Faced with the current development of robotics, existing legal norms may be inadequate to regulate the interaction between humans and intelligent robots with AI.

The European Parliament realized this inadequacy; on 16 February 2017, it passed a resolution (2015/2103 INL) with “recommendations to the Commission on Civil Law Rules on Robotics” [75].

In brief, with this act, the European Parliament invited the European Commission to draft and submit to the European legislature a proposal for a directive identifying general civil law provisions relating to the use of robots with AI, to be applied in the member states.

The resolution notes:

… that the potential for empowerment through the use of robotics is nuanced by a set of tensions or risks and should be seriously assessed from the point of view of human safety, health and security; freedom, privacy, integrity and dignity; self-determination and non-discrimination, and personal data protection ….

Because of these issues, the report advocated the establishment of a new European agency for robotics and artificial intelligence, a code of ethical conduct for robots, responsibility rules, and a legislative framework.

The resolution also had the effect of enabling and facilitating the enactment of regulations in the health sector, such as Regulation (EU) 2017/745 of the European Parliament and of the Council of 5 April 2017, subsequently amended with respect to the dates of application of some of its provisions, moving the effective date from 26 May 2020 to 26 May 2021, by Regulation (EU) 2020/561 of 23 April 2020.

The next step was the approval of Resolution 2020/2014 INL of 20 October 2020 (recommendations to the Commission on a civil liability regime for AI) [76].

Point 2 of the resolution urged the approval of a legislative framework common to member countries: “… a horizontal and harmonised legal framework based on common principles seems necessary to ensure legal clarity, to establish equal standards across the Union and to effectively protect our European values and citizens' rights ….”

The concerns about the apparent existence of a legislative vacuum are well represented in section 6 of the act:

… the complexity, connectivity, opacity, vulnerability, the capacity of being modified through updates, the capacity for self-learning and the potential autonomy of AI systems, as well as the multitude of actors involved represent nevertheless a significant challenge to the effectiveness of Union and national liability framework provisions; considers that specific and coordinated adjustments to the liability regimes are necessary to avoid a situation in which persons who suffer harm or whose property is damaged end up without compensation …

Europe is therefore very clear that it must address this issue in a serious manner, being called upon to provide answers that cannot wait long.

The willingness of the European Union to make a concrete commitment is not, however, in question, given the establishment of the European AI Alliance and the Technical Committee for High-Risk AI Systems (TCRAI-committee), which demonstrates how the institution is engaging in a dialogue not only interinstitutionally, but also with stakeholders.

The European AI Alliance is a participatory platform created with the aim of promoting discussion and collecting contributions from citizens, companies, and scholars on the topic of AI.

The initial purpose of the forum was to provide feedback to the group of 52 high-level experts on AI (AI HLEGs) appointed by the European Commission to assist in policy development, but as time has passed, the AI Alliance has become a true focal point in stakeholder-driven discussions of AI policy.

The Technical Committee for High-Risk AI Systems (TCRAI) has the function of supporting the European Commission in its periodic review under the European regulation and includes representatives of member states as well as a balanced selection of stakeholders.

One of the most delicate points on which the European institutions are most often called to provide an answer is the possible recognition of a legal status for robots equipped with AI, which would make them holders of rights and duties, including that of restoring any damage caused.

The need to design a specific legal space for the robot with AI arises from the observation that an android capable of making decisions independently and without external conditioning (“strong AI”) is not characterized as a product, or as a medical device, and even less as a tool.

In Italy, professional liability in healthcare is regulated under Law No. 24 of 2017 (called the Gelli-Bianco law).

This law's main objectives were to put a brake on the rampant phenomenon of defensive medicine and to limit healthcare litigation, providing greater protection for healthcare professionals and guaranteeing them greater protection under the law.

The new physiognomy of the culpable responsibility of healthcare professionals is now based on a detailed regulation of the guidelines, which identify the recommendations that tend to be binding for healthcare professions, and on the introduction, in the Penal Code, of a new article concerning the culpable responsibility for death or personal injuries in the healthcare field (art. 590-sexies), marked by the elimination of the gradation of guilt and the limitation of nonpunishability to only the unskillful conducts, provided that they are meeting the applicable guidelines [77].

In extreme synthesis, under the criminal law profile, the healthcare professional is liable, by way of fault, for death or personal injuries resulting from the exercise of medical-surgical activity in the following four cases:

1. If the event occurred because of negligence (even slight) or imprudence
2. If the event occurred because of negligence (even slight) due to inexperience when the concrete case is not governed by the recommendations of the guidelines or good clinical-assistance practices
3. If the event occurred due to negligence (even slight) from inexperience in the identification and choice of guidelines or good practices that are not appropriate to the specificity of the concrete case
4. If the event occurred due to serious fault from inexperience in the implementation of recommendations, guidelines, or good clinical-assistance practices that are appropriate, considering the degree of risk to be managed and the specific technical difficulties of the medical act [78]

On the other hand, from the civil point of view, the Gelli-Bianco law has established a double track, configuring a contractual responsibility of the healthcare facility (whether private or public) and a noncontractual responsibility of the healthcare professional, unless the latter has stipulated a contract with the patient.

The legislative intervention was justified by the desire to bring the responsibility of the healthcare professional within the scope of the rules of noncontractual responsibility regarding the burden of proof (in particular, the fault and causal link) and the limitation period (five years, different from the ten years provided for contractual responsibility) [79].

Another crucial innovation the Gelli-Bianco law introduced is represented by the centrality of the safety of care, understood as a fundamental component of healthcare and an essential element for the provision of high-quality services.

As evidence of the preeminent role the safety of healthcare plays, it should be noted that the law opens with a strong statement of intent on this issue: “Safety of care is a constitutive part of the right to health and is pursued in the interest of the individual and the community.” [80].

This strongly affirms that the right to health, in its personal and subjective dimension, can also be understood as a right to care that, although conditioned by limited financial resources, cannot be denied to individuals. This is a very important interpretative statement of principle, to which numerous innovations introduced by the law and operating on the level of prevention and risk management and implemented by public and private health and social-health facilities are related.

The quality and safety of care therefore become, under the Gelli-Bianco law, essential components in the provision of health services [81].

It is from this legal framework that a profound reflection on the use of robots in healthcare must begin: can widespread use of social and assistive robots in nursing care meet the need to provide safe health services to the community?

The certainty regarding the safety of the use of robots is still decidedly lacking at present.

Although encouraging safety standards have been achieved in the experimentation of robots used in the health sector, the definition of zero risk is far from being achieved, especially in view of the continuous progress in technological development, which provides us with increasingly intelligent and autonomous robots.

In view of these uncertainties, the existence of a solid legal framework, capable of establishing with certainty who should pay for any errors or damage caused by a robot, is of central importance.

With reference to civil law, if we try to apply the ordinary rules of civil liability to robots, we can come to three natural conclusions:

1. Robots, insofar as they do not have legal personality—having never acquired legal capacity, which, according to Italian law can only be acquired by human beings at the moment of birth—cannot be held personally liable for the damage they cause by act or omission
2. According to the rules currently in force, a specific responsibility is identifiable only in the head of a specific human agent to whom the damaging action the robot caused can be traced (for example the manufacturer or the programmer)
3. To establish liability, it is necessary that the agent could have foreseen and avoided the robot's harmful behavior

Within this legal context, which considers the robot as a mere tool, the doctor or nurse would be fully responsible for any damage the robot caused (a kind of strict liability).

This approach would be detrimental in terms of quality of healthcare, since it would represent the birth of a new form of defensive medicine: doctors and nurses would tend to avoid using robots as much as possible, since they would be responsible for the damages they caused to patients.

Moreover, the attribution of civil liability to the doctor for a robot's inadequate conduct, as much as it may be justified in view of the position of guarantee that the Italian Constitution and jurisprudence attribute to the doctor towards the patient, would be in clear contrast with the extra-contractual nature of the liability of the health professional as enshrined in Law 24/2017.

Therefore, the Italian regulatory system, as defined by the Gelli-Bianco law, is clearly inadequate to guarantee to the patient the fundamental right to compensation for damages caused by the new generation of robots, pushing, on the contrary, healthcare professionals to adopt defensive medicine behaviors, that is, abstaining from the use of robots.

The simplest solution, on which European legislation is also focusing, is represented by the recognition of a specific legal status for intelligent robots, which could be the prelude for a definition of a system of responsibility that would enable the coexistence of patient safety and a confident use of robots in healthcare [82].

Two opposing views are possible regarding the criminal liability of robots.

According to the first one, the robot should be understood as a simple object, and therefore not criminally responsible for any crimes it commits; instead, the programmer should be responsible.

However, at this point a problem of imputability would arise: if the robot is provided with decisional autonomy, is the programmer imputable? If so, is the responsibility intentional or negligent? According to the organic immedesimation theory, it would be intentional, since the action performed by the non-human agent is an extension of the human agent's will.

The reading of the responsibility of the robot as entirely ascribable to the designer or programmer could even take on paradoxical connotations if dropped into the Italian regulatory context. Article 111 of the Italian Penal Code states: “Whoever has determined to commit a crime a person who is not imputable, or not punishable because of a condition or personal quality, is liable for the crime committed by this person, and the penalty is increased....”

The robot would then be judged in the same way as minors who are not chargeable for a crime their parents have induced them to. Not only would the programmer or designer (and, to remain within the simile, the minor's parents) be held criminally responsible, but the penalty would be increased.

Such a provision, if applied with erroneous assumptions regarding the actual degree of self-determination of the automaton, would lead to legal distortions (in the case, for example, where it is erroneously assumed that the robot depends entirely on the designer, when, instead, it takes illegitimate actions on its own initiative).

According to the second view, the robot should be understood as a new subject of criminal law, criminally responsible.

Admitting this scenario, however, should entirely redefine the perimeters of the concepts of classical criminal law (concept of completeness, subjective capacity, action, etc.), to design a criminal context applicable to the world of robots.

Among the most fervent supporters of the second view, that robots are criminally prosecutable just like humans, is Israeli criminal lawyer Gabriel Hallevy.

In Hallevy's view, the constitutive elements of the crime can easily be applied to AI systems, which therefore must be considered fully chargeable subjects.

Regarding the objective element of the crime, intended as the whole of conduct, event and causal relationship between conduct and event, in fact, there are no elements that can exclude the attribution of this component of the crime to a robot.

In other words, a robot can be responsible for a fact identified by the legal system as criminally relevant. Consider the context of nursing robotics where a nurse robot causes a patient to fall to the ground, causing the patient to suffer a severe head injury that leads to death.

According to Hallevy, the subjective (or psychological) element of the crime can also be charged to a robot. Since many robots are able to store data from the outside world, to foresee the consequences of their actions, and even to put in place a conduct suitable for the achievement of a specific goal, the critic does not see any obstacle to the realization, in the AI of the machine, of a criminal intent, realisable in the form of negligence or general intent (a category that, for Hallevy, includes intention, knowledge, and recklessness).

In essence, therefore, Hallevy strongly questions the axiom of *machina delinquere (et puniri) non potest*, which he considers to be a mere metaphysical and anthropocentric prejudice, comparable to the scepticism that had accompanied the recognition of the criminal liability of corporations (*societas delinquere non potest*), which then crumbled in the face of its affirmation at common law.

Hallevy theorised three models of AI entity criminal liability:

1. The perpetration-via-another liability model
2. The natural-probable-consequence liability model
3. The direct liability model

The first model foresees an indirect responsibility of the human agent (builder, programmer, final user), while the second and third models foresee a primary responsibility of the robot, which could eventually be associated to a concomitant responsibility of the human [83]. There are essentially three main objections to Hallevy's theory.

First, many critics point out that robots cannot in any way be attributed the subjective element of the crime, since, although supported by what superficially may appear to be a capacity for self-determination, robots (even the most advanced ones) do not have the ability to set themselves selfish goals of behavior and to choose whether it is worth putting other people's legal goods at risk to achieve them.

Second, any penalties imposed on robots would be completely ineffective since they would not be able to fulfil their re-educational or deterrent function.

The third and final criticism has to do with the loss of a truly criminal meaning of a penalty imposed on a robot.

This is because a sanction aimed at AIs (unlike humans) essentially affects no one else but themselves, since, after being created, they undergo progressive autonomy, becoming free.

This implies that a robot, even if sanctioned, will not influence the behavior of any human being, and even if this were possible, in any case, humans could not influence the behavior of the artificial subject [84].

## 5. Conclusions

This paper attempted to illustrate the bioethical landscapes of robotic nursing.

Through a scoping review approach, we identified the most relevant scientific papers focusing on the ethical implications of nursing practice at the dawn of the fourth industrial revolution.

The limitations of the present study are mainly the omission of grey literature analysis and the relatively small number of articles that met the inclusion and exclusion criteria and were therefore studied in detail in order to propose an answer to the review questions. Given the scarcity of papers dealing with this topic in an organized and systematic way, and of rather rigid exclusion criteria, we indeed selected only 14 articles, which we nevertheless found to be sufficient to understand the state of the art of bioethics applied to robotic nursing.

To interpret in the most correct way the results of the research, we proposed an extended treatment of the ethical-philosophical context, within which the discussion arises, starting from Asimov's laws of the 1940s up to the contemporary theories of nursing robotics.

We also found it helpful to propose specific considerations regarding the healthcare and cultural context of Italian nursing, as well as to illustrate a brief overview of the medical-legal implications related to an extensive use of robots in nursing, again with a focus on the Italian reality.

Overall, based on our literature review, we can state that the ethical issues related to the use of robots in the context of nursing can no longer be ignored.

In fact, for some time now, the technologization of healthcare has overwhelmingly invaded the field of nursing, which must therefore resolve, as soon as possible, the ethical-legal issues related to the use of nursing robots.

These issues, in addition to the aspect of patient safety, concern the very concept of nursing care, whose basic theoretical models must necessarily be reviewed and updated.

Those who must play a proactive role in this process of adaptation of theoretical paradigms are the nurses, who, as custodians of nursing knowledge, are the only ones able to propose an effective system of human-machine integration.

However, according to our analysis of the experts' opinions, it seems that, at least for the time being, robots can only play a secondary role in the nursing process.

As a matter of fact, the conditions do not currently seem to exist for robots to enter the nursing care relationship, except in a mere communication role.

Regarding models of robot integration within nursing practice, the traditional models of NAC and CCVSD are being joined by new theoretical horizons, represented by the three currently most accredited models, the dance of living caring model (a synergistic fusion of NAC and CCVSD), the TRETON model, and the TCCN model.

These three approaches have in common the active involvement of the robot, which is valued as a tool to achieve the fullness of the therapeutic alliance between human nurse and patient.

However, these promising models of robot engagement are difficult to apply in practice in the absence of a clear definition of the legal framework for robot liability.

In fact, we have observed how a confused regulatory framework represents a highly favorable element for the tendency of healthcare professionals (including nurses) to feed a new frontier of defensive medicine, represented by abstention from the use of robots.

In conclusion, therefore, whatever the role of robots within nursing care is, we must seriously question ourselves on what ideal of care to set the nursing care of the robotic era, keeping in mind that the implementation of a project of human-robot collaboration in an ethical key cannot disregard a regulatory framework that defines as clearly as possible the responsibility profiles of the actors of the relationship, human and robot, in order to prevent attitudes of prevention by the nursing staff.

## Figures and Tables

**Figure 1:** PRISMA-ScR (preferred reporting for systematic reviews and meta-analyses extension for scoping reviews) flow diagram for study selection.

**Table 1:** The PCC framework (inclusion criteria).

	Main concept	Alternate keywords	Subject headings (MeSH)
Participants	—	—	—

Concept	Robots	Robot, Robotic, Robotics, Technology, Robotic Systems, Smart Systems, Automated Systems, Machines, Autonomous Systems, Humanoids, Humanoid Robotics, Robotic Technology	Robotics
	Ethical Issues	Ethical, Ethics, Ethical Implications, Moral Issues, Moral Implications, Dilemma, Dilemmas, Ethical Responsibility	Ethical issue/ethical issues/ethics/ethics, situational/issue, ethical/issues, ethical

Context	Nursing Care	Nursing, Assistive, Caregivers, Nursing Homes, Personal Care	Care, nursing/management, nursing care/nursing care/nursing care management

**Table 2:** Search strings used to search the Ovid Medline database.

*#*	Searches	Results
1	exp robotics/	30,140
2	robot^*∗*^.mp. [mp = title, abstract, original title, name of substance word, subject heading word, floating subheading word, keyword heading word, organism supplementary concept word, protocol supplementary concept word, rare disease supplementary concept word, unique identifier, synonyms]	40,095
3	robotic^*∗*^.mp. [mp = title, abstract, original title, name of substance word, subject heading word, floating subheading word, keyword heading word, organism supplementary concept word, protocol supplementary concept word, rare disease supplementary concept word, unique identifier, synonyms]	36,651
4	technology.mp. [mp = title, abstract, original title, name of substance word, subject heading word, floating subheading word, keyword heading word, organism supplementary concept word, protocol supplementary concept word, rare disease supplementary concept word, unique identifier, synonyms]	341,977
5	robotic system^*∗*^.mp. [mp = title, abstract, original title, name of substance word, subject heading word, floating subheading word, keyword heading word, organism supplementary concept word, protocol supplementary concept word, rare disease supplementary concept word, unique identifier, synonyms]	2,458
6	smart system^*∗*^.mp. [mp = title, abstract, original title, name of substance word, subject heading word, floating subheading word, keyword heading word, organism supplementary concept word, protocol supplementary concept word, rare disease supplementary concept word, unique identifier, synonyms]	184
7	automated system^*∗*^.mp. [mp = title, abstract, original title, name of substance word, subject heading word, floating subheading word, keyword heading word, organism supplementary concept word, protocol supplementary concept word, rare disease supplementary concept word, unique identifier, synonyms]	4,229
8	machine^*∗*^.mp. [mp = title, abstract, original title, name of substance word, subject heading word, floating subheading word, keyword heading word, organism supplementary concept word, protocol supplementary concept word, rare disease supplementary concept word, unique identifier, synonyms]	142,054
9	autonomous system^*∗*^.mp. [mp = title, abstract, original title, name of substance word, subject heading word, floating subheading word, keyword heading word, organism supplementary concept word, protocol supplementary concept word, rare disease supplementary concept word, unique identifier, synonyms]	293
10	humanoid^*∗*^.mp. [mp = title, abstract, original title, name of substance word, subject heading word, floating subheading word, keyword heading word, organism supplementary concept word, protocol supplementary concept word, rare disease supplementary concept word, unique identifier, synonyms]	571
11	robotic technology.mp. [mp = title, abstract, original title, name of substance word, subject heading word, floating subheading word, keyword heading word, organism supplementary concept word, protocol supplementary concept word, rare disease supplementary concept word, unique identifier, synonyms]	808
12	1 OR 2 OR 3 OR 4 OR 5 OR 6 OR 7 OR 8 OR 9 OR 10 OR 11	515,875

13	exp ethical issue/	148,641
14	ethical issue^*∗*^.mp. [mp = title, abstract, original title, name of substance word, subject heading word, floating subheading word, keyword heading word, organism supplementary concept word, protocol supplementary concept word, rare disease supplementary concept word, unique identifier, synonyms]	1,1142
15	ethic^*∗*^.mp. [mp = title, abstract, original title, name of substance word, subject heading word, floating subheading word, keyword heading word, organism supplementary concept word, protocol supplementary concept word, rare disease supplementary concept word, unique identifier, synonyms]	202,109
16	ethical implication^*∗*^.mp. [mp = title, abstract, original title, name of substance word, subject heading word, floating subheading word, keyword heading word, organism supplementary concept word, protocol supplementary concept word, rare disease supplementary concept word, unique identifier, synonyms]	1,856
17	moral issue^*∗*^.mp. [mp = title, abstract, original title, name of substance word, subject heading word, floating subheading word, keyword heading word, organism supplementary concept word, protocol supplementary concept word, rare disease supplementary concept word, unique identifier, synonyms]	619
18	moral implication^*∗*^.mp. [mp = title, abstract, original title, name of substance word, subject heading word, floating subheading word, keyword heading word, organism supplementary concept word, protocol supplementary concept word, rare disease supplementary concept word, unique identifier, synonyms]	185
19	dilemma^*∗*^.mp. [mp = title, abstract, original title, name of substance word, subject heading word, floating subheading word, keyword heading word, organism supplementary concept word, protocol supplementary concept word, rare disease supplementary concept word, unique identifier, synonyms]	32,769
20	Ethical Responsibility^*∗*^.mp. [mp = title, abstract, original title, name of substance word, subject heading word, floating subheading word, keyword heading word, organism supplementary concept word, protocol supplementary concept word, rare disease supplementary concept word, unique identifier, synonyms]	692
21	13 OR 14 OR 15 OR 16 OR 17 OR 18 OR 19 OR 20	263,936

22	exp care, nursing/	136,709
23	nurs^*∗*^.mp. [mp = title, abstract, original title, name of substance word, subject heading word, floating subheading word, keyword heading word, organism supplementary concept word, protocol supplementary concept word, rare disease supplementary concept word, unique identifier, synonyms]	700,325
24	assistive.mp. [mp = title, abstract, original title, name of substance word, subject heading word, floating subheading word, keyword heading word, organism supplementary concept word, protocol supplementary concept word, rare disease supplementary concept word, unique identifier, synonyms]	5,687
25	caregivers.mp. [mp = title, abstract, original title, name of substance word, subject heading word, floating subheading word, keyword heading word, organism supplementary concept word, protocol supplementary concept word, rare disease supplementary concept word, unique identifier, synonyms]	62,370
26	nursing home^*∗*^.mp. [mp = title, abstract, original title, name of substance word, subject heading word, floating subheading word, keyword heading word, organism supplementary concept word, protocol supplementary concept word, rare disease supplementary concept word, unique identifier, synonyms]	44,788
27	personal care.mp. [mp = title, abstract, original title, name of substance word, subject heading word, floating subheading word, keyword heading word, organism supplementary concept word, protocol supplementary concept word, rare disease supplementary concept word, unique identifier, synonyms]	4,676
28	22 OR 23 OR 24 OR 25 OR 26 OR 27 OR 28	75,4617

	12 AND 26 AND 36	**930**

**Table 3:** Summary of the key findings obtained from the review of the 14 selected articles.

Author(s)	Title	Author(s)' country	Year of publication	Type of article and study design (if applicable)	Aims	Key findings that relate to the scoping review question
*Descriptive articles with literature review*						
Fuji et al. [19]	Discussion of nursing robots' capability and ethical issues	Japan-USA	2014	Traditional literature review	Discussing the ethical implications associated with the use of robots in the nursing setting	The widespread use of robots in nursing is an unstoppable and rapidly evolving phenomenon, so it is necessary to identify a way for humans and robots to interact effectively.

Metzler et al. [22]	Could robots become authentic companions in nursing care?	USA	2016	Traditional literature review	Understanding whether robots can effectively fit within the nursing relationship	Robots may not currently be eligible to take an active role in the caregiving relationship.

Barcaro [23]	Ethics of care and robot caregivers	Slovenia-Italy	2018	Traditional literature review	Exploring new ways of caring for humans using robotic assistants considering the ethical issues/questions of respecting the human dignity	It is essential that we implement collaboration between human nurses and assistive and social robots, with a view to making the most of robotic resources, which are often superior to human ones.

Bulfin et al. [26]	Anne Boykin Institute for the advancement of caring in nursing use of robots to complement caring relationships in nursing position paper	USA	2019	Position paper	Giving an interpretive reading relative to the role of robots in assisting the nursing staff	Nurses must have an active and proactive role in defining the role of robots in nursing care.

Grobbel et al. [27]	Designing nursing care practices complemented by robots: ethical implications and application of caring frameworks	USA-Netherlands	2019	Traditional literature review	Exploring the ethical framework of the care-centred value-sensitive design (CCVSD) and the role that robots can play within it	Nurses must take the lead and define how robots should be used in clinical practice, to protect the sacred nurse-patient relationship.

Robson [24]	Intelligent machines, care work and the nature of practical reasoning	UK	2019	Traditional literature review	Exploring issues of the moral status and limitations of machines in the context of care based on the principles of MacIntyre's philosophy	Robots, regardless of the level of technological advancement, cannot be moral agents, and thus cannot care.
Christoforou et al. [20]	The upcoming role for nursing and assistive robotics: opportunities and challenges ahead	Cyprus	2020	Survey research. The study was conducted through the administration of a questionnaire to 115 students and alumni of the Department of Nursing, Faculty of Health Sciences, at Cyprus University of Technology (CUT) in September 2019.	Providing an overview of today's nursing and care robotics landscape, highlighting the benefits associated with the adoption of such solutions in clinical practice, and identifying the major challenges facing the healthcare system in the future	The interviewees expressed a marked inclination to enter a nursing context characterised by a collaboration between men and robots, especially considering the possibility of delegating to the latter the less clinical and more boring tasks related to nursing care.

Servaty et al. [21]	Implementation of robotic devices in nursing care. Barriers and facilitators: an integrative review	Germany	2020	Integrative review	Identifying the main barriers to and facilitators of the implementation of robotic systems in nursing	The facilitating elements identified were adapting robot functions to the needs of users; individuals' positive attitude towards technology; positive feelings towards the devices; acceptance of end users; active involvement of healthcare teamwork; considering technology as a source of support for nurses and physicians; and a clear identification of roles, responsibilities, and expectations.

Yew [28]	Trust in and ethical design of carebots: the case for ethics of care	Singapore	2020	Traditional literature review	Illustrating the challenges associated with the ethical use of assistive and social robots in healthcare	Tronto's vision of care ethics, based on the principles of attentiveness to needs, responsibility, competence, and responsiveness, is the best model for integrating assistive and social robots into nursing care.

Stokes and Palmer [25]	Artificial intelligence and robotics in nursing: ethics of caring as a guide to dividing tasks between AI and humans	USA	2020	Traditional literature review	Understanding the most appropriate role that robots can play in the context of nursing care, taking care ethics theory as a basic ethical reference	Artificial intelligence, at least for the foreseeable future, does not possess the prerequisites to be able to care for the patient in the central sense of nursing ethics and caregiving, although it can fill minor tasks.

*Articles proposing an ethical theory to facilitate the integration of robots into nursing care*						
Tanioka [29]	The development of the transactive relationship theory of nursing (TRETON): a nursing engagement model for persons and humanoid nursing robots	Japan	2017	Traditional literature review	Identifying a theoretical framework in which to incorporate human and robot collaboration in nursing care	The theoretical approach resulting from the fusion of the nursing as care (NAC) approach and the TCCN (technological competency as caring in nursing) model is represented by the TRETON.
Tanioka et al. [30]	Recommended design and direction of development for humanoid nursing robot's perspective from nursing researchers					

Locsin and Ito [31]	Can humanoid nurse robots replace human nurses?	Japan	2018	Traditional literature review	Describing issues about humanoid robots and their influences on the discipline and professional practice of nursing	The TCCN theory represents the ideal model to enable effective integration of robots within nursing care.

Schoenhofer et al. [32]	Engaging robots as nursing partners in caring: nursing as caring meets care-centred value-sensitive design	USA-Netherlands	2019	Traditional literature review	Finding a methodological approach adaptable to robotic nursing through the conjugation of the CCVSD model and the NAC model.	The theoretical approach resulting from the fusion of the CCVSD model and the NAC model is represented by the dance of living caring model, which is based on three principles: Intentional knowing of persons as caring, respecting and valuing persons as caring, and hearing and responding to calls for caring.

## Data Availability

The data used to support the findings of this study are included within the article.
